The article "A Random Walk with Restart Model Based on Common Neighbors for Predicting the Clinical Drug Combinations on Coronary Heart Disease" was retracted in 2023. Reasons: signs of a paper mill; suspected computer-generated content; unreliable results or conclusions; lack of ethics approval or compliance.

# A Random Walk with Restart Model Based on Common Neighbors for Predicting the Clinical Drug Combinations on Coronary Heart Disease

**DOI:** 10.1155/2021/4597391

**Published:** 2021-12-08

**Authors:** Yushi Che, Wei Cheng, Yiqiao Wang, Dong Chen

**Affiliations:** ^1^School of Management, Beijing University of Chinese Medicine, Beijing 100029, China; ^2^Xingzhi College, Zhejiang Normal University, Jinhua, Zhejiang 321000, China

## Abstract

As the approaching of the clinical big data era, the prediction of whether drugs can be used in combination in clinical practice is a fundamental problem in the analysis of medical data. Compared with high-throughput screening, it is more cost-effective to treat this problem as a link prediction problem and predict by algorithms. Inspired by the rule of combined clinical medication, a new computational model is proposed. The drug-drug combination was predicted by combining the number of adjacent complete subgraphs shared by the two points with the restart random walk algorithm. The model is based on the semisupervised random walk algorithm, and the same neighborhood is used to improve the random walk with restart (CN-RWR). The algorithm can effectively improve the prediction performance and assign a score to any combination of drugs. To fairly compare the predictive performance of the improved model with that of the random walk with restart model (RWR), a cross-validation of the two models on the same drug data was performed. The AUROC of CN-RWR and RWR under the LOOCV validation framework is 0.9741 and 0.9586, respectively, and the improved model results are more reliable. In addition, the top 3 predictive drug combinations have been approved by the public. The new model is expected that this model can be extended to predict the use of combination drugs for other diseases to find combinations of drugs with potential clinical benefits.

## 1. Introduction

Recently, due to the aging society, accelerating process of urbanization, and prevalence of unhealthy lifestyle, the number of coronary heart disease risk factor exposure has increased significantly. Global health indicators show that coronary heart disease (CHD) has the highest prevalence rate among all cardiovascular diseases. CHD's mortality rate is the leading cause of death in middle-income countries [1, 2]. Because CHD is a disease with many complications, the condition of patients with CHD is complex. Doctors tend to treat patients with multiple medications, also known as drug combinations, to reduce symptoms of CHD and its complications. In such cases, drug combination is more advantageous than single-drug treatment [3, 4]. In order to ensure the scientific and rational use of drug combinations, researchers often use high-throughput methods to explore the possibility of drug combinations. In the scientific trial screening of the efficacy and rationality of drug combinations, the high-throughput drug-screening technologies which conduct large-scale experiments on cultured human cell line panels are used generally [5]. While one significant disadvantage of the high-throughput drug-screening technologies is that only one protein is being screened at a time, lowering the number of total potential hits as compared to alternative screening methods. At the same time, it will inevitably consume a lot of time and resources in the process of goals vague experiments. In addition, the clinical drug combination in the field of coronary heart disease drug therapy compared with drug trials in the lab will be more complex. Some of the complex prescriptions taken by doctors are the result of years of experience or careful consideration. As a result, drug use is more flexible in clinical practice, and many combinations of effective drugs may be overlooked in laboratory trials. Therefore, there is a pressing need for a time-saving and resource-saving approach that can predict the actual clinical drug combinations.

Now, because of the prevalence of predictive algorithms, researchers applied machine learning models to predict drug combinations. So far, some methods predict drug combinations based on drug property similarity or by link prediction. Traditional link prediction methods analyse the network's topological structure and evaluate the similarity of node pairs in the network, based on the intuition that node pairs with high similarity are more likely to be linked. Lorrain et al. [6] proposed a method for computing node similarity based on their common neighbors. In other words, the similarity between two points is equal to the number of their common neighbors. This index is relatively simple, but in the network with high aggregation coefficient, its prediction effect can even surpass some more complex algorithms. Zhou et al. [7] introduced another method based on degree information. It takes into account the resource propagation between two indirectly linked nodes via their common neighbors. In addition, they also proposed a path-based semilocal similarity index, which converts the network relationship from a graph with circles to a tree form and constructs a similarity function by comparing the number of paths with lengths of 2 and 3. On the basis of this index, it is extended to be a global index based on path similarity, the Katz index. Francois et al. [8] predicted links with the similarity of random walk sequences. The basic idea of this algorithm is to traverse a graph from one or a series of vertices. In the process of random walk, there are different probability walk to the neighbor node of the previous state node or random jump to any vertex on the graph. The probability distribution after walking is iterative as the input of the next walk. The stable probability distribution after convergence is the similarity between nodes in the graph.

Although the above four link prediction methods are not particularly new, they provide inspiration for follow-up studies. Some researchers have proposed link prediction with a better prediction effect based on the traditional link prediction method and have achieved great success in the field of drug combination prediction. For example, the random walk with restart model gives scores of node-to-node connections based on degree information [9]. Moreover, RWR has been successfully applied to data mining applications, such as ranking [10], link prediction [11, 12], and community detection [13]. On the application of the algorithm in predicting drug combination, Di et al. [14] put forward a method, called termed prioritization of candidate drugs, that prioritizes the cancer drug candidate by applying a global network propagation algorithm to a drug functional similarity network. The correlation of drugs based on mRNA and microRNA pathways and the correlation between each channel activity built a drug functional similarity network based on mRNA and microRNA pathways and determine the degree of drug similarity in the similar network. Rohani et al. [15] introduced their algorithm, called NDD, which utilizes the neural network model along with similarity selection and fusion methods to take advantage of nonlinear analysis and professional feature extraction to improve the prediction accuracy of drug-drug interaction. The models proposed by these studies have significantly improved performance compared with previous models. However, the drugs' chemical properties and drug targets were used for prediction as data sources of these studies. In the real world, the doctor has more autonomy when they prescribe. They will take into account a patient's special and complex condition. Doctors will use drug combinations flexibly, especially when treating diseases with many complications. It will make the kinds of the actual drug combinations more than the predicted kinds of the drug combination based on pharmacological and chemical properties. Thus, the results of these studies may differ from the drug combinations that use in real-world clinical.

For similarity selection, finding the regular patterns of drug combinations used by clinicians in the real world to predict drug combinations is a more direct way. Shtar et al. [16] treat the drug-drug interaction problem as a link prediction problem and propose two methods based on neural networks and factor propagation on graph nodes, adjacency matrix factorization (AMF), and adjacency matrix factorization with propagation (AMFP). They evaluate the effect of drug-drug interactions, create an ensemble-based classifier using AMF, AMFP, and current link prediction methods, and achieve a good performance. From the study, it is testified that drug combinations can be predicted by the combination law of drugs. The form of data used in the study is similar to drug combinations in prescription. The artificial neural network algorithm (ANN) was used in Shtar's study. One of the problems of ANN is the unexplained behavior of the network. ANN can produce a probing solution, but it does not provide an explanation, which reduces trust in the network. Based on the above research results, it is significant to explore that a model is appropriate for predicting drug combinations in the clinic.

In clinical medication, we find that in drug combinations, if two drugs have more adjacent complete subgraphs (i.e., two third-order complete subgraphs are adjacent), it is more likely for them to have an edge. In other words, if two drugs have more commonly combined drugs, they are more likely to be combined. As shown in Figure 1, *i* and *j* denote two drugs. If they have more commonly combined drugs, drugs *i* and *j* have a higher probability to be combined.

Compared with drug network based on pharmacological and chemical properties, the more relationship between the two nodes needs to be captured in the real drug network. We consider the topological nature of the drug network, and this method can reveal some special rules of the drug combination in the clinic. Therefore, we evaluate drug similarity by the drug network's topological property and treat drug combination as a link prediction problem. We explore an improved random walk with restart (RWR) algorithm based on common neighbors, CN-RWR. We construct a drug network in which each node denotes a drug and each edge denotes a combination. The random walk with restart algorithm is conducted by analyzing the possible common complete subgraphs formed by two nodes and using them as transition probabilities. In this way, the connection between each node and other nodes will have a link probability. Thus, it can predict the combination probability of two drugs in the treatment of coronary heart disease. In the implementation of the algorithm, we study the value of the restart probability of RWR on common neighbors. Moreover, our model achieves a significantly higher AUROC, as validated by cross-validation. Case studies validate the effectiveness and potential of our CN-RWR.

The remainder of the paper is organized as follows. In Section 2, materials and methods are introduced.  Section 3 summarizes the results and discussion, and Section 4 illustrates the conclusions and future work.

## 2. Materials and Methods

### 2.1. Datasets and Evaluation Metric

Since this study is based on a predictive analysis of actual clinical use of combination drugs, we study the CHD drugs which have been used to treat the patient in the clinic medical records. The experimental datasets were obtained from the drug combinations of outpatient prescriptions for patients with coronary heart disease in a grade-A tertiary hospital from 2014 to 2016. Due to the protection of hospital and patient privacy information, the name of the hospital and patient is not listed. The definition of CHD drugs comes from the CHD Medication Guidelines (version 2) which refer to the evidence quality and recommendations in the guidelines published by the European Society of Cardiology (ESC), American College of Cardiology (ACC), and American Heart Association (AHA). Finally, we collect 212,402 prescriptions and 57 drugs. Among them, 1,341 drug combinations have been applied clinically and are marked as positive examples. The rest combinations are marked as negative examples.

Due to uncertain thresholds, we employ AUROC [17] as the evaluation metric. AUROC is not affected by the list length or threshold, so it is applied to evaluate the performance of binary classifiers. AUROC denotes the area under the ROC curve [18], and its value varies between 0 and 1. A higher AUC value means better performance.

### 2.2. CN-RWR Overview

We define an undirected graph *G*=(*V*, *E*) in which each node denotes a drug for CHD. For any two nodes, they are connected by an edge if and only if the corresponding two drugs have appeared in the same prescription. So rules of the relationship between the two drugs are as follows:

(1) $$\begin{array}{c} \left\{\begin{array}{c} \left(i,j\right)=1|i,j\text{ in the same prescription,}\\ \left(i,j\right)=0|i.j\text{ did not appear in either prescription.} \end{array}\right. \end{array}$$

Based on the adjacency matrix constructed above, we carry out the random walk on the graph. A random walk on a graph is a transition from a given vertex to a randomly selected neighbor at each step. We define a node set {*v*_1_, *v*_2_,…, *v*_*n*_} as the initial set of a Markov chain {*s*_1_, *s*_2_,…, *s*_*n*_}. Markov chain's transition probability is defined as a conditional probability *P*(*u*, *v*)=*P*(*s*_*t*+1_=*v|s*_*t*_=*u*), which denotes the probability of random walk arriving at node *v* at time *t* + 1, while at time *t*, it is at node *u*. For any *v* ∈ *V*, the marginal probability ∑_*v*∈*V*_*P*(*u*, *v*) is always 1. Thus, we obtain a transition matrix *P* ∈ *ℝ*^|*V*|×|*V*|^.

In graph *G*, *P*(*u*, *v*) denotes the transition probability of a random walk from *u* to v:

(2) $$\begin{array}{c} P\left(u,v\right)=\frac{\Gamma \left(u\right)\cap \Gamma \left(v\right)}{\Gamma \left(u\right)\cap \Gamma \left(V/u\right)}, \end{array}$$

where Γ(*u*)∩Γ(*v*) denotes the number of *u* and *v*′*s* common neighbors. Γ(*u*)∩Γ(*V*/*u*) is the number of *u* and all other nodes' common neighbors, which excludes self-combination. We use the inner product of adjacency matrices to compute the value of Γ(*u*)∩Γ(*v*):

(3) $$\begin{array}{c} \Gamma \left(u\right)\cap \Gamma \left(v\right)=\sum_{n=1}^{\left|V\right|}\left(i,n\right)\left(j,n\right)\left(n\in V;i,j\in A\right), \end{array}$$

where *A* is the adjacency matrix. Adjacency matrix *A* denotes the combinations of drugs used in prescriptions. *A* is square matrix. The elements in the matrix are defined as the combination of the drug in row *i* and the drug in column *j*. If two drugs appear in one prescription at the same time, the corresponding element is equal to 1. Otherwise, it is equal to 0.

We define a vector *r*_*t*_ ∈ *ℝ*^|*V*|×1^. Its *i*-th element starts random walking at time *t* and its state at time *t* + 1 is

(4) $$\begin{array}{c} r_{t+1}=P^{T}r_{t}. \end{array}$$

We adopt random walk with restart, so the above equation is rewritten as

(5) $$\begin{array}{c} r_{t+1}=cP^{T}r_{t}+\left(1-c\right)r_{0}, \end{array}$$

where *r*_0_ ∈ *ℝ*^|*V*|×1^ is the initial probability distribution. Its *i*-th element is 1, and the rest are 0.1 − *c* is the restart probability, where 0 ≤ *c* ≤ 1. To study the restart probability 1 − c's impact on the classifier's performance, we change the value of 1 − *c* from 0.05 to 0.95, and the spacing between 1 − *c* is adjusted by 0.05, obtaining the AUROC scores and standard deviations based on LOOCV of 19 different parameter values were calculated.

The random walking starts from an initial node *v*_*i*_ and visits other nodes according to the above transition probability. Assuming that it arrives at node *u*_*j*_ at time *t* + 1, the probability of arrival by random walk is *c*, and the probability of restart is 1 − *c*. After multiple iterations, random walk probabilities converge, and *r*_*t*_ + 1 − *r*_*t*_ is smaller than any arbitrary value. We set this threshold to 10^−6^ which is often adopted in other studies [19, 20]. When random walk converges, we obtain a matrix *Z*={*z*_*ij*_}_|*V*|×|*V*|_, where each element *z*_*ij*_ denotes the stable probability of random walk from node *v*_*i*_ to *v*_*j*_. In other words, when the *i*-th element of *r*_*0*_ is 1, element *j*'s stable probability $z_{ij}=\underset{t⟶\infty }{\lim}r_{t}$. The value of *z*_*ij*_ denotes the probability of combining drugs *i* and *j* by analyzing the common neighbors of the two drugs. Graph *G* is unweighted and undirected, so the matrix *Z* is symmetric. Thus, we obtain the scores of all drug combinations *S*={*s*_ij_}_|*V*|×|*V*|_:

(6) $$\begin{array}{c} s_{ij}=\left\{\begin{array}{cc} z_{ij}+z_{ji}, & i\neq j,\\ 0, & i=j. \end{array}\right. \end{array}$$

This algorithm can give the score of any two drugs' combination. A higher score denotes a more probable combination, so in clinical or experimental trials, these combinations with higher scores can be validated first, thus greatly reducing the labor and cost of verifying the combination.

## 3. Results and Discussion

### 3.1. Experimental Setup

Based on the Jupyter Notebook platform, Pandas and NumPy were used in the experiment to preprocess the data. Excel was used to build the adjacency matrix of drug combinations. The new model based on common neighbors and the classical RWR model were written and run on MATLAB. The evaluation indexes, AUC, were chosen to evaluate the performance of two models. In order to improve the accuracy of the results, we adopt leave-one-out cross-validation (LOOCV).

### 3.2. Cross-Validation and Restart Probability

LOOCV is widely used when the data are limited. Although we have a great number of prescription data, there are fewer kinds of drugs. LOOCV is more applicable to a small dataset. And it generally performs very well with regard to MSE and bias [21]. It focuses on an accurate estimate of model performance more than the computational cost of the method. Therefore, we use LOOCV to evaluate the performance of various methods.

We split the drug combinations whose corresponding value in the adjacency matrix is 1 into a training set and a test set and choose the combinations with value 0 in the adjacency matrix as candidate examples. The trained model predicts the scores of every example in the test set and candidate set. LOOCV is selected for the division of training set and test set in both our model (CN-RWR) and comparative model (RWR). In each run, it takes a positive example (a drug combination that has been applied clinically) as the test set and the rest (other drug combinations which have been applied clinically) as the training set. All nonpositive examples (other possible drug combinations) are candidate examples. After obtaining all examples' scores, we take all positive examples as the test set and compare its scores with those of candidate examples. The performance based on LOOCV with different 1 − *c* values is shown in Figure 2after determining the method of cross-validation, and in order to make the comparison results of the prediction performance of the two models, we assign the same restart probability for the restart random walk and our improved algorithm.

The bar and line charts denote the AUROC values and standard deviations, respectively, when varying the restart probability. As can be intuitively seen from the figure, as the restart probability of the restart random walk increases, the AUROC score gradually decreases. We hope that the prediction performance of our model is relatively optimal. When the restart probability is 0.05, the performance of the model is best. The value of SE is lower in different values of 1 − *c*, and the AUC's value is highest. Therefore, we selected the restart random walk model when the parameter 1 − *c* was 0.05 to carry out the model comparison of the prediction drug combination.

### 3.3. Model Comparison

The random walk with restart model based on neighbor nodes and the random walk with restart model were used to predict drug combinations in the constructed network, and the prediction performance of the two models was compared. For a fair comparison, we use the same data of drug combination of clinical to compare two models.

In the prediction studies, the performance measurement is an essential task. It can count on an AUC-ROC curve. The AUC-ROC curve is also written as AUROC (area under the receiver operating characteristics). ROC is a curve of probability. The ROC curve is plotted with sensitivity against specificity where sensitivity is on the *y*-axis and (1-specificity) is on the *x*-axis. Sensitivity, also known as true positive rate (TPR), represents the ratio of true positive to all positive in the positive class predicted by the classifier. 1-Specificity, also known as false-positive rate (FPR), represents the ratio of false positive to all negative in the positive class predicted by the classifier. Formulas of TPR and FPR are as follows:

(7) $$\begin{array}{c} \text{TPR}=\frac{\text{true positive}}{\text{true positive}+\text{false negative}},\\ \text{FPR}=\frac{\text{false positive}}{\text{false positive}+\text{true negative}}. \end{array}$$

The value of AUC is the area under the ROCs' curve of the graph. ROCs' curves are drawn, and values of AUC are calculated on MATLAB.

ROCs' curves of two models and values of AUC are shown in Figure 3. The AUC values predicted by each model were in the range from 0.5 to 1. The prediction accuracy of two models was better than random guessing and had predictive value. Besides, the CN-RWR values of AUC were 0.9741, and the AUROC value of RWR is about 0.9586. The results indicate that the performance of the CN-RWR model was better in the drugs combination network, and the forecast accuracy was improved significantly. Although the random walk model can be used to predict the combination of drugs for clinical use, the CN-RWR is more reliable because it takes into account the special rule of the drugs' network.

### 3.4. Case Study

This paper is based on actual outpatient data and combines RWR and common neighbors to find new drug combinations. In the search for combination drugs, we selected some drug combinations as the validation of the model's ability to predict drug combinations, that is, we selected the top 19 drug combinations with the highest predicted scores and summarized their clinical use frequency of combined drugs in Table 1.

Based on the predicted results of the CN-RWR model, we can obtain the combined scores of any two drugs in the drug network. In Table 1, the top three drug combinations: atorvastatin-aspirin, clopidogrel bisulfate-aspirin, and clopidogrel bisulfate-atorvastatin are shown. They all had combined scores of 0.041681915. The result shows that the drug combinations of these three groups were equally likely in the prediction. And they are more likely to be used by doctors. From the actual prescription data, we know that the times of using Atorvastatin and Aspirin are up to 30678 times. The times of using Bisulfate and Aspirin are 30146. The times of using Clopidogrel Bisulfate and Atorvastatin are 16527. Doctors who treat coronary heart disease often use these combination drugs in practical treatment. The prediction result is confirmed. The model is suitable for predicting drug combinations in the real world. In addition, the top 3 drug combinations have been shown to be effective in treating coronary artery disease. Among them, Aspirin and Clopidogrel Bisulfate are recognized worldwide as an effective combination for coronary heart disease. Nabeel et al. [22] even successfully create a new polypill with atorvastatin calcium, clopidogrel bisulfate, and aspirin.

In 16 other drug combinations, their combined scores were 0.041505407. They were used in clinical with the lowest frequency of 5417 times and the highest frequency of 32215 times. It indicates that these drug combinations have been used frequently in clinical practice. The drug combinations predicted by the new model have been used by doctors for clinical.

Ninety-five percent of the top 19 drug combinations given by CN-RWR have the top 10% frequency in clinical medication. In other words, drug combinations with high scores are often applied clinically. Judging whether drug combinations are used in practice based on the clinical combination scores obtained from the CN-RWR model is important in understanding the clinical use of combination drugs.

## 4. Conclusion and Future Work

This paper introduces CN-RWR, a generalization of random walk with restart based on common neighbors. Compared with the classical RWR model which calculates the transition probability based on degree information, a new model (CN-RWR) was proposed that the transition probability was calculated based on the possible common complete subgraph formed by the two nodes in the paper. Our results show that the prediction performance of the CN-RWR model is better than the RWR model by the prediction performance measurement. Besides, we have collected data from outpatient prescriptions and used the CN-RWR algorithm to predict the clinical drug combinations on coronary heart disease. The CN-RWR model can successfully predict some of the common drug combinations. Our work summary is shown in Table 2.

In addition, in many studies, the pharmacological and chemical properties of drugs are used to predict drug combinations. In the real world, however, the doctor has more autonomy when they prescribe. They will be using drug combinations according to the actual situation of patients. It will make the kinds of the actual drug combinations more than the predicted kinds of the drug combination based on pharmacological and chemical properties. Thus, we use the drugs' network topology based on the common neighbor node number of similarities between the two nodes to simulate the drug combinations in the clinic. It makes the predicted results more similar to the drug combinations in the real world.

To sum up, this paper is a realistic perspective to predict the actual drug combinations used in clinical practice. Based on the drug combinations used by doctors, we constructed a drug relationship network and compared the prediction performance of the improved restart random walk model and the restart random walk model of neighbor nodes based on the cross-validation of the retention method. The experimental results show that our model has a strong prediction ability. In the case study, we obtained some meaningful information about the clinical use of combination drugs from the predicted results of the CN-RWR model. And we find that the real combination network is a highly clustered network, which might be related to doctors' treatment experience in clinical. Therefore, future work is needed to explore the generalizability of our model to other diseases. We hope that other researchers who have the conditions to study prescription drugs for other diseases can try to use our model to conduct further studies on the current situation of combined drug use in real life.

In future studies, we will deepen the drugs network level, add the weighting information, and introduce demographic factors of patients, such as the age and gender, in order to broaden the scope of the study and improve the prediction accuracy.

## Figures and Tables

**Figure 1:** *i* and *j* denote two drugs. Other nodes denote drugs that are used in combination with drug *i* and drug *j*. The solid lines indicate drug combinations used in a prescription. The dotted line indicates the possibility of two medications being combined. Two drugs are more likely to be combined if they share more commonly combined drugs.

**Figure 2:** The LOOCV performance when varying the restart probability.

**Figure 3:** The ROCs of CN-RWR and RWR models with LOOCV.

**Table 1:** Case study of drug combination prediction.

Drug 1	Drug 2	Score	Frequency of drug combination
Atorvastatin	Aspirin	0.041681915	30678
Clopidogrel bisulfate	Aspirin	0.041681915	30146
Clopidogrel bisulfate	Atorvastatin	0.041681915	16527
Amlodipine besylate	Aspirin	0.041505407	12150
Amlodipine besylate	Atorvastatin	0.041505407	6050
Isosorbide mononitrate	Aspirin	0.041505407	32215
Isosorbide mononitrate	Atorvastatin	0.041505407	15226
Bisoprolol fumarate	Aspirin	0.041505407	15007
Bisoprolol fumarate	Atorvastatin	0.041505407	6688
Metoprolol succinate	Aspirin	0.041505407	26114
Metoprolol succinate	Atorvastatin	0.041505407	10606
Metoprolol tartrate	Aspirin	0.041505407	13254
Metoprolol tartrate	Atorvastatin	0.041505407	6060
Clopidogrel bisulfate	Amlodipine besylate	0.041505407	4964
Clopidogrel bisulfate	Isosorbide mononitrate	0.041505407	19706
Clopidogrel bisulfate	Bisoprolol fumarate	0.041505407	5417
Clopidogrel bisulfate	Metoprolol succinate	0.041505407	14779
Clopidogrel bisulfate	Metoprolol tartrate	0.041505407	6314
Rosuvastatin	Aspirin	0.041505407	29655

**Table 2:** Work summary.

Evaluation tools	MATLAB
Performance metrics	SE, ROCs' curve, and values of AUC
Case studies	The clinical drug combinations on coronary heart disease
Deployment strategy	Data management of the outpatient prescription: data collection, data preprocessing
	Model learning: design CN-RWR model, model selection (RWR), training, parameter selection (c in leave-one-out cross-validation (LOOCV))
	Model verification: simulation-based testing
Advantages	The prediction algorithm in this study was based on the topological properties of a drug combinations network in the real world and it makes the predicted results more similar to the drug combinations of the real world Our model performance is better than the traditional one
Disadvantages	The predictive performance of the model can be further improved

## Data Availability

The data used to support the findings of this study are available from the corresponding author upon request.
